# Severe Dextran-Induced Anaphylactic Shock during Induction of Hypertension-Hypervolemia-Hemodilution Therapy following Subarachnoid Hemorrhage

**DOI:** 10.1155/2015/967560

**Published:** 2015-06-11

**Authors:** Tohru Shiratori, Atsushi Sato, Masao Fukuzawa, Naoko Kondo, Shogo Tanno

**Affiliations:** ^1^Division of Intensive Care Unit, Ina Central Hospital, 1313-1 Koshiroukubo, Ina, Nagano 396-8555, Japan; ^2^Department of Neurosurgery, Ina Central Hospital, 1313-1 Koshiroukubo, Ina, Nagano 396-8555, Japan; ^3^Department of Dermatology, Ina Central Hospital, 1313-1 Koshiroukubo, Ina, Nagano 396-8555, Japan; ^4^Department of Anesthesiology, Ina Central Hospital, 1313-1 Koshiroukubo, Ina, Nagano 396-8555, Japan; ^5^Department of Emergency Medicine, Ina Central Hospital, 1313-1 Koshiroukubo, Ina, Nagano 396-8555, Japan

## Abstract

Dextran is a colloid effective for volume expansion; however, a possible side effect of its use is anaphylaxis. Dextran-induced anaphylactoid reaction (DIAR) is a rare but severe complication, with a small dose of dextran solution sufficient to induce anaphylaxis. An 86-year-old female who underwent clipping for a ruptured cerebral aneurysm was admitted to the intensive care unit. Prophylactic hypertension-hypervolemia-hemodilution therapy was induced for cerebral vasospasm following a subarachnoid hemorrhage. The patient went into severe shock after administration of dextran for volume expansion, and dextran administration was immediately discontinued. The volume administered at that time was only 0.8 mL at the most. After fluid resuscitation with a crystalloid solution, circulatory status began to recover. However, cerebral vasospasm occurred and the patient's neurological condition deteriorated. Five weeks after the shock, she was diagnosed with hypersensitivity to dextran by a skin test. When severe hypotension occurs after dextran administration, appropriate treatments for shock should be performed immediately with discontinuation of dextran solution. Although colloid administration is recommended in some guidelines and researches, it is necessary to consider concerning the indication for volume expansion as well as the risk of colloid administration.

## 1. Introduction

Dextran is a polysaccharide that is frequently used for volume expansion. Possible side effects of dextran infusion include allergic reactions. Anaphylaxis in response to dextran administration has been recognized as rare but life-threatening complication [1, 2]. Symptoms of severe dextran-induced anaphylactic reaction (DIAR) include bronchospasm, severe hypotension, and cardiorespiratory arrest [1, 3, 4].

In a retrospective survey in Sweden for the period from 1970 to 1979, the incidence of fatal DIAR was 0.003% due to dextran 40, which has a molecular weight of 40,000 daltons, and 0.004% due to dextran 70, with a molecular weight of 70,000 daltons [1]. A prospective study for the period of 1981–1986 showed that the incidence of severe DIAR was 0.12% in 5,747 patients undergoing obstetric and gynecologic surgery and to whom dextran 70 solution was administered [3]. The incidence of DIAR in stroke patients has not been investigated.

Most reactions occur within a few minutes after the beginning of dextran solution infusion [4]. Even a small dose of dextran solution can induce anaphylactic shock [1, 3]. Most people have low titers of dextran-reactive antibody (DRA), and serious DIAR usually occurs in patients with high DRA titers [2]. Appropriate treatment should be initiated rapidly when DIAR is suspected.

## 2. Case Presentation

An 86-year-old woman was admitted to our hospital because of severe headache and vomiting. She had a history of abdominal total hysterectomy when in her 50s. She had no previous history of allergy to foods or drugs. She had been prescribed benidipine hydrochloride for hypertension, raloxifene hydrochloride for osteoporosis, donepezil hydrochloride for dementia, and sodium ferrous citrate for iron deficiency anemia by her family physician.

On admission, Glasgow Coma Scale was E1V2M4, blood pressure was 224/102 mmHg, and the pulse rate was 69 beats/min. Her pupils were round and equally sized at 3 mm, and her respiratory condition was stable.

Emergent head computed tomography (CT) showed subarachnoid hemorrhage (SAH) with associated large sylvian fissure hematoma extending to the basilar cistern. CT angiography showed rupture of an aneurysm of the middle cerebral artery. She was classified as grade 4 by Hunt and Kosnik's classification and grade 3 by the modified Fisher CT rating scale. Clipping for the ruptured aneurysm was performed on the day of admission to prevent early rebleeding.

On postoperative day 1, she was mechanically ventilated in the intensive care unit using 40% oxygen, and her vital signs were stable. Propofol, ozagrel sodium, and cefazolin sodium were administered intravenously without any problems. Postoperative CT revealed no signs of rebleeding in the immediate vicinity of the ruptured aneurysm. Prophylactic treatment for cerebral vasospasm using hypertension-hypervolemia-hemodilution therapy (triple-H therapy) was induced. The administration of crystalloid solution minimized the development of hypovolemia and reduced the hematocrit level from 37.4% to 28.6%. Colloid solution was additionally administered in order to maintain a central venous pressure greater than 8 mmHg.

The infusion of 10% dextran 40 solution was initiated at a rate of 10 mL/hr. Prior to dextran infusion, blood pressure was 114/64 mmHg, the heart rate was 76 beats/min, and SpO2 was 100%.

Approximately 5 min after initiation of dextran infusion, systolic blood pressure suddenly dropped to 40 mmHg, and the pulse rate increased to 140 beats/min. The patient's face, chest, abdomen, and extremities became flushed and warm. The level of SpO2 remained stable at 100%. Auscultation revealed normal vesicular sound with no rales or crackles. An electrocardiogram showed tachycardia with no change in the ST segment.

Infusion of dextran solution was discontinued immediately. 500 mL sodium acetate solution was administered rapidly and crystalloid administration was continued at a rate of 500 mL/hr. 20 min after the initiation of the shock, systolic blood pressure was restored to 70 mmHg. Continuous infusion of 0.3% dopamine was started peripherally at a rate of 10 mL/hr. Echocardiography revealed normal heart structure compatible with a hyperdynamic state. Peripheral vascular resistance was predicted to be low. Administration of 0.05 mg noradrenaline improved systolic blood pressure, which increased to above 80 mmHg. One g methylprednisolone sodium succinate was also administered. Approximately 40 min after the initiation of the shock, systolic blood pressure rose to above 100 mmHg and the crystalloid administration rate was set at that of 100 mL/hr. While the patient was in shock status, 100% oxygen was administered temporarily. After the recovery from hypotension, the level of oxygen concentration was gradually decreased to that of 40%. While the patient was in shock, the level of SpO2 was kept at 100%. After these treatments, systolic blood pressure was maintained within the range of 130 mmHg to 160 mmHg with continuous dopamine infusion.

On postoperative day 7, CT revealed cerebral artery spasm and widespread cerebral ischemia in the right cerebral hemisphere with extensive brain swelling. Emergency decompressive hemicraniectomy was performed. Three weeks following hemicraniectomy, cranioplasty was performed and a ventriculoperitoneal shunt was placed. Although the postoperative course was uneventful, the patient's consciousness did not recover.

Five weeks after the shock, we performed a skin test with undiluted 10% dextran solution instead of an examination to detect DRAs.

The patient had been prescribed 3 L oxygen/minute via a face mask for mild congestive heart failure. Before skin test, blood pressure was 102/63 mmHg, the heart rate was 66 beats/min, and SpO2 was 99%. Skin prick test was negative. Approximately 15 min following the skin prick test, intradermal test was conducted with 0.025 mL undiluted 10% dextran solution. Approximately 30 min following the intradermal test, the patient developed a wheezy cough with flares and diffuse wheals on her face and extremities. Blood pressure decreased to 89/58 mmHg, the heart rate increased to 120 beats/min, and SpO2 decreased to 89%. Face mask oxygen was increased to 5 L/minute. Following administration of 200 mL crystalloid solution with 100 mg hydrocortisone and 50 mL of 20% albumin solution, systolic blood pressure recovered to values above 100 mmHg.

The results of the test showed that the patient was hypersensitive to dextran. It was assumed that the patient had suffered a severe anaphylactic reaction to dextran during the induction of the triple-H therapy.

Five months after admission, the patient was discharged to a rehabilitation hospital.

## 3. Discussion

The initial strategy for treating ruptured aneurysm is to prevent rebleeding. Surgical clipping is the definite treatment for ruptured aneurysms. The second target of treatment is to prevent or control cerebral vasospasm. Cerebral infarction due to cerebral vasospasm after SAH may lead to neurological deterioration [5–8]. Early surgery also permits early treatment for cerebral vasospasm with triple-H therapy when a ruptured aneurysmal sac is separated from the cerebral circulation [5].

Treatment for cerebral vasospasm relies on increasing blood pressure, cardiac output, and blood volume in order to maintain cerebral blood flow through spastic arteries in which the capacity of autoregulation is impaired. While recent researches show less clinical evidence in the triple-H therapy to require normovolemia instead of hypervolemia [5–7], early clinical response to induced hypertension and volume expansion predicts improved outcome in patients with vasospasm after SAH [8]. Triple-H therapy should be induced carefully to reduce the risk of complications.

SAH patients in triple-H therapy require volume expansion with crystalloid or colloid solution. Artificial colloids typically available include dextran and hydroxyethyl starch (HES) that are both widely used drugs for volume expansion [9].

Anaphylactic reaction to dextran is rare, but dextran can induce life-threatening adverse reactions known as DIAR, characterized by bronchospasm, severe hypotension, and cardiovascular collapse [1, 3, 4].

Severe DIAR is an immune complex mediated anaphylactic reaction classified as type III [2]. IgG-DRA is involved in the reaction [4].

DRAs are assumed to be induced by dextran polysaccharides that are derived from dextran contaminants in sugar, dextran in the gastrointestinal tract, dextran in dental plaque, and microbial polysaccharides of pneumococci,* Streptococci*,* Salmonella*, and* Lactobacilli* [1, 2, 10]. The antibody production rate by dextran tends to increase when the molecular weight of dextran is above 90,000 daltons [11]. Although dextran 40 is classified as a small molecule, it can cause a severe anaphylactic reaction [1, 4].

DRA exists at low titers in most people. High DRA titers have been detected in blood samples from patients with severe DIAR. Elevated DRA titers are associated with severe DIAR [1, 2, 9, 12].

Dextran 1, which has a molecular weight of 1,000 daltons, acts as a hapten and inhibits type III allergic reactions due to DRA, which prevents DIAR development. Although the risk of a fatal reaction cannot be completely eliminated by preadministration of dextran 1 in case the patient has a high level of DRA, preadministration of dextran 1 can decrease the incidence of severe DIAR [4, 10, 13–15].

In addition to dextran, HES is also used as a colloid solution for volume expansion. Although there are several case reports on HES-induced anaphylactic reactions [16–19], the incidence of such reactions to HES is extremely low compared with dextran [9, 20, 21]. While DRAs are found in most adults, HES-reactive antibodies are extremely rare [20, 21]. HES is a synthetic polymer derived from amylopectin, a waxy starch of maze. The reason for the low incidence of antibodies to HES is that the structure of HES resembles that of glycogen [20, 21]. Although HES may induce dilution of coagulation factors, HES can be administered instead of dextran in cases where tight hemostasis is completed during operation [22].

Recently, U.S. Food and Drug Administration (FDA) has recommended not to use HES solutions in critically ill adult patients because of the risk of increased mortality and renal injury requiring renal replacement therapy. However, renal injury was not evident in which HES solutions were administered for a short period within seven days according to FDA-analysis in a review of randomized controlled trials [23]. When using HES solutions, the period of HES administration should be limited within seven days and renal function monitoring is necessary.

The development of anaphylactic shock during post-SAH triple-H therapy induction is considered to be ill-timed. According to research reports on animal models [24–29], the direct action of anaphylactic mediators on the cerebral arterial system results in cerebral ischemia and brain injury. The decrease in cerebral blood flow is greater than what would be expected from the level of severity of arterial hypotension, which is attributed to the rapid and direct action of anaphylactic mediators on cerebral vessels [24, 25]. Even though blood pressure and cardiac output recover following anaphylactic shock, there is a risk of continued cerebral blood flow deterioration [26]. In addition, mast cell activation by anaphylaxis causes a substantial release of vasoactive inflammatory cytokines. Mast cells resident within the cerebral microvasculature act on the basal membrane and damage the blood-brain barrier, resulting in brain edema [24, 27, 28]. When anaphylactic shock occurs in patients suffering from SAH, it is important to take special notice of harmful effects due to anaphylactic shock on cerebral circulation.

The diagnosis of drug allergy is often based on history alone, which is an unreliable indicator of true hypersensitivity [30]. The methods that allow the definitive diagnosis of anaphylaxis include a complete clinical history, clinical manifestations,* in vivo* tests, and some* in vitro* biological tests [31]. Skin tests are the most widely used methods to confirm or exclude sensitization of drugs. Skin tests should be performed 4–6 weeks after the reaction [30, 31].

Although reliable skin test procedures including skin test concentrations for diagnosing drug hypersensitivity are available for some drugs, those for colloids are not presented. Many drugs are undiluted for skin prick test and diluted to 1/10 for intradermal test. Symptoms of skin tests may severely progress in some cases to bronchospasm, hypotension, and anaphylactic shock [30]. Diluted colloid solution should be used for secure intradermal test in critically ill patients who have presented severe anaphylactic symptoms.

When skin tests are not available in cases of poor outcome such as death,* in vitro* biological tests are helpful [32]. Biological tests are also useful for the patients who have the possibility of severe hypersensitivity [31–33].

Consecutive blood measurements of tryptase, which is released from mast cell and has a longer half-life than histamine, are also effective for confirming the occurrence of anaphylaxis [31–33].

Flow cytometry-assisted basophil activation test (BAT) can be utilized in the diagnosis of drug hypersensitivity [31, 34]. However, BAT is an expensive and technically difficult procedure. The recommended time interval between the anaphylactic reaction and BAT test is twelve months [34], which is longer than skin test [31]. Although BAT is the developing diagnostic method for anaphylaxis, it is safe compared with* in vivo* tests. BAT is supposed to be a promising diagnostic method for patients with severe anaphylactic reaction [31, 34].

Initial treatments for anaphylactic shock are extremely important. Guidelines recommend that epinephrine injection, supplemental oxygen, fluid resuscitation, and cardiopulmonary resuscitation should be initiated without delay [33, 35]. Epinephrine is used as a vasoconstrictor in the treatment of anaphylaxis, since prompt epinephrine use prevents the escalation of mediator release in anaphylaxis [35]. Fox et al. observed cerebral blood flow in a patient suffering from anaphylaxis. They reported that the increase of cerebral blood flow following epinephrine administration occurred before complete recovery of arterial blood pressure [36]. Norepinephrine is a vasoconstrictor commonly used to treat hypotension. However, there is a possibility that norepinephrine deteriorates post-SAH cerebral vasospasm in spite of high blood pressure [37]. Although there have been several case reports of DIAR for which epinephrine was not administered [10, 12, 38], epinephrine should have been administered as the first-line vasoactive agent in our case instead of norepinephrine. Supplemental high flow oxygen should be administered while a patient is in shock and 20 mL/kg crystalloid solution should be administered for fluid resuscitation enough to recover from severe hypotension [33, 35]. If hypotension continues, further crystalloid administration may be required [33].

Anaphylaxis must be considered as a possible cause in any case of hypotension [33]. When the patient went into shock, we had little confidence that only a small volume of dextran could cause severe anaphylaxis. However, we suspected anaphylaxis because of the redness of the whole body at onset. If hypotension occurs immediately after initiation of dextran infusion, discontinuation of dextran infusion is critical, since the severity of anaphylaxis increases if dextran infusion is continued as a fluid resuscitation for hypotension. It should be recognized that only a small volume of dextran is sufficient to induce anaphylaxis [1, 10]. Some guidelines and researches recommend the use of colloid solution for fluid resuscitation [35, 39]. Careful consideration is necessary concerning the risk of anaphylaxis due to colloids when administering colloid solutions for volume expansion in critical care patients.

## 4. Conclusion

In SAH-patients administered colloid solutions for volume expansion, it is important to become aware of and address the complication of colloid solutions, including anaphylaxis. Anaphylactic shock due to colloid used for volume expansion is life-threatening.

In order to recognize the occurrence of DIAR as early as possible, careful observation of the skin and checking of vital signs are necessary when administering dextran solution for the first time. It is critical to discontinue dextran infusion immediately in order to avoid administering the dextran solution as a volume expander after the shock.

When using colloids for post-SAH triple-H therapy, it is also necessary to consider concerning the indication for volume expansion as well as the risk of colloid administration.

Intradermal test should be conducted with diluted concentration in critically ill patients.

When the definitive diagnosis of drug hypersensitivity is required,* in vitro* biological test may be helpful in patients suspected to have severe drug hypersensitivity since allergic symptoms can progress.
